The article "Symmetric Deformable Registration via Learning a Pseudomean for MR Brain Images" was published in 2021. Journal: J Healthc Eng.

# Symmetric Deformable Registration via Learning a Pseudomean for MR Brain Images

**DOI:** 10.1155/2021/5520196

**Published:** 2021-04-23

**Authors:** Xiaodan Sui, Yuanjie Zheng, Yunlong He, Weikuan Jia

**Affiliations:** ^1^School of Information Science and Engineering, Shandong Normal University, Jinan 250358, China; ^2^Key Lab of Intelligent Computing and Information Security in Universities of Shandong, Shandong Provincial Key Laboratory for Novel Distributed Computer Software Technology, Institute of Biomedical Sciences, Shandong Normal University, Jinan 250358, China; ^3^INSA Lyon, University of Lyon, CNRS, Inserm, Villeurbanne 69621, Cedex, France

## Abstract

Image registration is a fundamental task in medical imaging analysis, which is commonly used during image-guided interventions and data fusion. In this paper, we present a deep learning architecture to symmetrically learn and predict the deformation field between a pair of images in an unsupervised fashion. To achieve this, we design a deep regression network to predict a deformation field that can be used to align the template-subject image pair. Specifically, instead of estimating the single deformation pathway to align the images, herein, we predict two halfway deformations, which can move the original template and subject into a pseudomean space simultaneously. Therefore, we train a symmetric registration network (S-Net) in this paper. By using a symmetric strategy, the registration can be more accurate and robust particularly on the images with large anatomical variations. Moreover, the smoothness of the deformation is also significantly improved. Experimental results have demonstrated that the trained model can directly predict the symmetric deformations on new image pairs from different databases, consistently producing accurate and robust registration results.

## 1. Introduction

Computer models have become a usable method for solving biomedical engineering and are applied to the analysis and measurement of data in the biomedical field (e.g., material mechanical behavior measurement [1–4], medical image segmentation [5, 6], and registration [7–9]). Deformable image registration aims to align subject images onto a template space by gradually optimizing the spatial transformation fields consisting of voxel-to-voxel correspondences between template and subject images [10]. Deformable registration is a key procedure in clinical applications such as population analysis, longitudinal data analysis, and image-guided intervention. Many image registration algorithms have been proposed and applied to various imaging analysis tasks [7–9, 11–16]. Conventional registration algorithms achieve the task via typical optimization, which can be classified into either intensity-based registration [11–13] or feature-based registration [14–16]. In these methods, the deformation field is obtained by iteratively optimizing the image similarity metric with a smoothness regularization constraint.

The article "Symmetric Deformable Registration via Learning a Pseudomean for MR Brain Images" was published in 2021. Journal: J Healthc Eng.

In recent years, deep learning has been widely applied in medical image analysis [17, 18]. And deep-learning-based registration methods have shown promising performance especially for efficiency, as the computational time can be significantly reduced from minutes to seconds. Since the ground-truth deformations are difficult to obtain in practice, some semisupervised [19] and unsupervised learning strategies [20–22] are more popular currently. Specifically, the spatial transformation network (STN) [23] is leveraged in the deep-learning-based registration framework so that the loss can be defined directly on the image similarity, instead of using ground-truth deformations as supervised information. When the model is well trained, in the application stage, the transformation field can be estimated for unseen image pairs, without the need for iterative optimization. Therefore, deep-learning-based registration is more flexible in real clinical use. Additionally, to further improve the registration accuracy, multiscale strategy [24, 25], diffeomorphic strategy [26], and inverse-consistent properties [27] are also incorporated in the deep-learning-based registration framework.

However, for the aforementioned registration algorithms, it is difficult to accurately register the images with large anatomical variation, and the smoothness is even difficult to preserve and constrain for large deformation. Thus, it is essential to develop an algorithm, which can effectively register the images with large anatomical variations and, meanwhile, keep the transformation field smooth, so that the topology can be well preserved. In addition, symmetric diffeomorphic registration has achieved better performance overall, which estimates symmetrical deformation pathway from two objects (template and subject) to the intermediate point instead of a single pathway from template to subject [13, 28]. Inspired by these methods, we hope to add a symmetric image registration strategy to the unsupervised model.

In this paper, we further investigate the deep-learning-based registration by considering the symmetric property. We propose a symmetric registration network (S-Net) by simultaneously aligning the subject and template images to an intermediate space, i.e., the pseudomean space. Specifically, instead of establishing the voxel-to-voxel correspondences in one pathway, i.e., from template space to subject space, we move the template and subject images symmetrically, until they meet in the pseudomean space. In this space, the image similarity is maximized. The main contribution of this work can be summarized as follows:

1. We propose a symmetric registration network that can register images in the dual direction simultaneously. In this framework, the pseudomean space can be automatically learned by using the symmetric constraint without any supervised guidance.
2. The symmetric property allows for estimating two short deformation pathways instead of directly estimating a long deformation pathway. It is more effective to register images with large anatomical variations. The final registration result can be more accurate and smoother.
3. Under the symmetric framework, we can directly obtain the forward (register subject to template) and backward (register subject to template) transformation fields by using the trained S-Net. Therefore, the inverse consistency can be achieved without introducing any additional model or strategy.

The article "Symmetric Deformable Registration via Learning a Pseudomean for MR Brain Images" was published in 2021. Journal: J Healthc Eng.

## 2. Materials and Methods

The S-Net is trained in an unsupervised manner based on the proposed symmetric way. As shown in Figure 1, the input of the network is a pair of template image *I*^*T*^ and subject image *I*^*S*^, together with their difference map. Instead of directly estimating the deformation field *ϕ* to register the subject to template, we make the training of the registration network symmetric, i.e., the template and subject image both deform until reaching their pseudomean space. Two deformation pathways will be estimated under this framework: (1) *ϕ*^*T*^ is the deformation pathway between template and pseudomean space and (2) *ϕ*^*S*^ is the deformation pathway between subject and pseudomean space.

Mathematically, the optimization of symmetric registration can be formulated by minimizing the image dissimilarity in the pseudomean space:

(1) $$\begin{array}{c} F\left(I^{S},I^{T},\phi^{S},\;\phi^{T}\right)=M\left(T\left(I^{S},\phi^{S}\right),T\left(I^{T},\phi^{T}\right)\right)+\lambda R\left(\phi^{S},\;\phi^{T}\right), \end{array}$$

where *𝒯*(*∗*, *∗*) is a deformation operation that can warp *I* by *ϕ* and *M* is the dissimilarity between the deformed subject image *I*^*S*^(*ϕ*^*S*^) and deformed template image *I*^*T*^(*ϕ*^*T*^). *R* is a regularization term to constrain the smoothness of two symmetric deformations *ϕ*^*T*^ and *ϕ*^*S*^. *λ* is a weight to balance the registration accuracy and deformation smoothness. In the training of the deformable registration network S-Net, *M* and *R* are used to define the loss function and *𝒯* is the spatial transformation network [23] used to spatially transform the image based on the estimated transformation field. The details of training the symmetric registration network S-Net will be described in Section 2.1.

The article "Symmetric Deformable Registration via Learning a Pseudomean for MR Brain Images" was published in 2021. Journal: J Healthc Eng.

In the testing stage, giving an unseen image pair and their difference maps, we can get their symmetric deformations *ϕ*^*S*^ and *ϕ*^*T*^. As shown in Figure 2, the final symmetric registration results can be obtained by composing the two predicted deformation pathways: the forward deformation can be formulated as *F*=*ϕ*^*T*^∘(*ϕ*^*S*^)^−1^, which can register the subject to template. The backward deformation can be formulated as *F*^−1^=*ϕ*^*S*^∘(*ϕ*^*T*^)^−1^ which can register the template to the subject. *ϕ*^*T*^∘(*ϕ*^*S*^)^−1^ is the inverse field of *ϕ*^*S*^∘(*ϕ*^*T*^)^−1^, and “∘” denotes the composition operator [28].

### 2.1. Symmetric Network Design

For symmetric registration, the pseudomean is an intermediate space on the image manifold, and the distance between the pseudomean and the template should equal that between the pseudomean and the subject. Therefore, for each location/voxel, the deformation magnitudes of *ϕ*^*T*^ and *ϕ*^*S*^ should be equal to each other, while the direction should be opposite. Thus, during the training, the output of the network is only *ϕ*^*T*^, and we can set *ϕ*^*S*^=−*ϕ*^*T*^. There are two advantages to using this symmetric setting. (1) The large local deformation can be more effectively estimated since we shorten the deformation pathway during registration. (2) We can easily keep the inverse consistency without introducing any additional constraint.

The S-Net was designed based on the network architecture designed in VoxelMorph [20], which is lighter than the original U-Net [6] by reducing the redundant connections to adapt to the analysis of 3D images. The network output is the halfway deformation *ϕ*^*T*^. Since we do not have the ground-truth deformations, herein, we apply the unsupervised training strategy [20–22]. Specifically, a spatial transformer network [23] provides a fully differentiable spatial transformation layer *𝒯* that can transform the input image *I* by the output deformation *ϕ*, which is the output of the S-Net. Specifically, we use the trilinear interpolation in STN, and the operation *𝒯* can be formulated as

(2) $$\begin{array}{c} T\left(I,\phi \right)=\sum_{v\in N\left(u+\phi \left(u\right)\right)}I\left(v\right)\;\prod_{d\in \left\{x,y,z\right\}}\left(1-\left|u_{d}+\phi \left(u_{d}\right)-v_{d}\right|\right), \end{array}$$

where *u*=[*x*, *y*, *z*] is the voxel coordinate, *N*(*u*+*ϕ*(*u*)) is the eight neighbor voxels of *u*+*ϕ*(*u*) in *I*, and *d* indicates three directions in 3D space. With STN, the loss defined by the image similarity can backpropagate to the S-Net, and the registration network can be trained in an unsupervised manner.

The article "Symmetric Deformable Registration via Learning a Pseudomean for MR Brain Images" was published in 2021. Journal: J Healthc Eng.

### 2.2. Loss Definition

#### 2.2.1. Symmetric Similarity Loss

The similarity loss of the registration task is used to evaluate the registration accuracy, and here, we define the similarity loss by SSD. Conventionally, the subject image should be warped to the template space by the output deformation field, and the loss is calculated in the template space. For the symmetric registration network, we define the similarity loss in the pseudomean space to penalize the symmetric property. Mathematically, it can be formulated as

(3) $$\begin{array}{c} {ℒ}_{\text{Sim}}^{\text{sym}}=T\left(I^{S},\phi^{S}\right)-T{\left(I^{T},\phi^{T}\right)}_{2}^{2}\text{,}\;\phi^{S}=-\phi^{T}. \end{array}$$

By minimizing the symmetric similarity loss ℒ_Sim_^sym^, the template and subject image will gradually register with each other, until they reach their pseudomean space. To further enhance the symmetric constraints and registration accuracy, we also define the similarity loss in both template and subject image space:

(4) $$\begin{array}{c} {ℒ}_{\text{Sim}}^{I^{S}⟶I^{T}}=T\left(I^{S},\phi^{S}\circ {\left(\phi^{T}\right)}^{-1}\right)-I_{2}^{T2},\\ {ℒ}_{\text{Sim}}^{I^{T}⟶I^{S}}=T\left(I^{T},\phi^{T}\circ {\left(\phi^{S}\right)}^{-1}\right)-I_{2}^{S2}, \end{array}$$

where *ϕ*^*S*^∘(*ϕ*^*T*^)^−1^ indicates the *forward* deformation pathway, which can transform the subject image to the template space, while *ϕ*^*T*^∘(*ϕ*^*S*^)^−1^ indicates the *backward* deformation pathway, which can transform the template image to the subject space. It worth noting that the output of the S-Net is the halfway deformation *ϕ*^*T*^, and the symmetric loss ℒ_Sim_^sym^ defined in the pseudomean space can well preserve the symmetric property, while ℒ_Sim_^*I*^*S*^⟶*I*^*T*^^ and ℒ_Sim_^*I*^*T*^⟶*I*^*S*^^ defined in the end image space can make the registration accurate. Therefore, the whole symmetric similarity loss can be summarized as ℒ_Sim_=ℒ_Sim_^sym^+ℒ_Sim_^*I*^*S*^⟶*I*^*T*^^+ℒ_Sim_^*I*^*T*^⟶*I*^*S*^^.

#### 2.2.2. Field Regularization Loss

The regularization loss is used to constrain the smoothness of the estimated deformation field *ϕ*^*T*^, which is important to preserve the topology. In S-Net, this regularization loss is only defined on *ϕ*^*T*^ (output of the network). The smoothness of *ϕ*^*S*^ can be automatically constrained since *ϕ*^*S*^=−*ϕ*^*T*^. In our work, three kinds of regularization loss, i.e., Laplace smoothness, zero constraint, and antifolds constraint, are used to penalize the smoothness.

(1) Laplace smoothness *L*_Laplace_: constraining the smoothness of the field *ϕ*^*T*^, which is defined as

(5) $$\begin{array}{c} {ℒ}_{\text{Laplace}}=\sum_{u}\nabla^{2}\phi^{T}{\left(u\right)}_{2}^{2}, \end{array}$$

where ∇^2^*ϕ*(*u*) is the second derivative of the field *ϕ*^*T*^(*u*) at the voxel *u*.

(2) Zero constraint: modifying the displacement value for avoiding unreasonable large deformations:

(6) $$\begin{array}{c} {ℒ}_{\text{Zero}}=\sum_{u}\phi^{T}{\left(u\right)}_{2}^{2}. \end{array}$$

(3) Antifolds constraint: adding an antifolds constraint [27] in the loss function to further enhance the smoothness constraint, avoiding folds, or crossing in the final deformation:

(7) $$\begin{array}{c} {ℒ}_{\text{Anti}}=\sum_{u}R\left(\nabla \phi^{T}\left(u\right)+1\right), \end{array}$$

where ∇*ϕ*(*u*) is the gradient of the displacement map and the term *R*(∇*ϕ*(*u*)+1) is an index function to penalize the gradient of the deformation field with folds. If *Q* ≤ 0, *R*(*Q*)=|*Q*|, and *R*(*Q*)=0, for otherwise.

The article "Symmetric Deformable Registration via Learning a Pseudomean for MR Brain Images" was published in 2021. Journal: J Healthc Eng.

The final loss function for training the S-Net is

(8) $$\begin{array}{c} {ℒ}_{\text{Loss}}={ℒ}_{\text{Sim}}+{ℒ}_{\text{Reg}}={ℒ}_{\text{Sim}}^{\text{sym}}+{ℒ}_{\text{Sim}}^{I^{S}⟶I^{T}}+{ℒ}_{\text{Sim}}^{I^{T}⟶I^{S}}+\alpha {ℒ}_{\text{Lap}}+\beta {ℒ}_{\text{Zero}}+\gamma {ℒ}_{\text{Anti}}, \end{array}$$

where *α*, *β*, and *γ* are used to balance the weight for each term. In this work, we set *α*=1 and *γ*=100 in our experiment. For zero constraint term *L*_Zero_, we set the weight *β* a small value as *β*=0.01, since the large value may influence the accuracy when estimating the large deformations.

### 2.3. Implementation and Training

The S-Net is implemented in Keras and trained on an NVIDIA Tesla V100 GPUs with 32 GB of video memory. The network is trained by using the Adam strategy [29]. We use four public databases, i.e., LONI LPBA40 [30], IBSR18 (https://www.nitrc.org/projects/ibsr), CUMC12 [31], and MGH10 [32] in our experiments. All images were preprocessed by using a standard pipeline, including skull stripping, resampling, and affine registration to the MNI152 template [33] by using FLIRT [34]. After preprocessing, the data are with the same size 192 × 224 × 192 (voxel size 1 mm × 1 mm × 1 mm).

We used 30 subjects from LONI LPBA40 dataset as the training data, and 30 × 30=900 image pairs can be derived. The remaining 10 images were used as the testing data, where 10 × 9=90 image pairs can be derived. The other three datasets are also used as the testing data to further evaluate the effectiveness of the proposed method, and we have 18 × 17=306 image pairs from IBSR18,  12 × 11=132 image pairs from CUMC12, and 10 × 9=90 image pairs from MGH10. For more effective training, we trained S-Net in two stages. First, the network was pretrained with a small dataset, where we chose one image as template and all the remaining images as subject. In this scenario, we totally have 1 × 30=30 image pairs for training. The network was trained for 200 iterations per image pair at a learning rate of 1*e* − 4. Then, we draw each two images as a template and subject pair, and we totally have 30 × 30=900 image pairs for further training the S-Net. 20 epochs were trained in this scenario, the learning rate is set to 1*e* − 5, with a decay weight of 0.5 for every 2 epochs.

The article "Symmetric Deformable Registration via Learning a Pseudomean for MR Brain Images" was published in 2021. Journal: J Healthc Eng.

## 3. Results

We have compared our results with three state-of-the-art registration methods, namely, D. Demons [12], SyN [13], and VoxelMorph [20]. Demons and SyN are typical deformable registration methods enforced successfully for the medical image registration task, and VoxelMorph is a learning-based framework that defines registration as a learnable parametric function. We conducted the experiment and measured the registration accuracy based on the volumetric overlap of brain ROIs. The overall registration accuracy was computed in the form of a Dice Similarity Coefficient (DSC) score Dice(*R*_*i*_^*S*^,  *R*_*i*_^*T*^)=(2*R*_*i*_^*S*^∩*R*_*i*_^*T*^)/(|*R*_*i*_^*S*^|+| *R*_*i*_^*T*^|), for each ROI, with *R*_*i*_^*S*^ and  *R*_*i*_^*T*^ being the corresponding anatomical regions *i* in the subject and template image. Additionally, we also evaluate the smoothness of the transformation map by using the Jacobian determinant *J*_*ϕ*_(*u*). Transformation map is considered smoothness when *J*_*ϕ*_(*u*) > 0, where *J*_*ϕ*_(*u*)=|*Dϕ*^−1^(*u*)| [35]. And, the overall folds of the estimated displacement map are defined in |{*u* : *J*_*ϕ*_(*u*) < 0}|.

The results of DSC scores and runtimes are shown in Table 1 compared with those state-of-the-art registration methods (Demons, SyN, and VoxelMorph). The results show that the proposed method performs significantly better than VoxelMorph (learning-based method without using a symmetric training manner). For some datasets, our approach even outperforms SyN, which was among the state-of-the-art brain image registration algorithms and only took about 3.6 seconds to register two brain volume data efficiently. Those learning-based methods, compared with the regular scenario, have shorter runtime, and also performance hardly deteriorates. In Table 2, we present the folds in the estimated displacement maps of the proposed method and the baseline method. The results show that the displacement maps are estimated by the proposed symmetric registration network smoothness more than by the model without asymmetric strategy in most cases by a large margin.

The article "Symmetric Deformable Registration via Learning a Pseudomean for MR Brain Images" was published in 2021. Journal: J Healthc Eng.

The respective results and intermediate results are also shown in Figures 3(b)–3(e) (final warped template image, middle warped subject image, middle warped template image, and final warped subject image, respectively). The S-Net works better than directly registering images in a single pathway: not only the registration accuracy but also the smoothness is also largely improved. This indicates that the proposed symmetric training strategy can effectively estimate large local deformations and the estimated field is smoother.

It is worth noting that S-Net achieves image registration tasks in an unsupervised end-to-end fashion by using an image similarity metric for optimization so that the training of this S-Net does not require the known deformation field, which is difficult to obtain for medical image registration. Furthermore, we have also evaluated our framework for the number of folds with the traditional registration method and single-direction deep-learning-based registration method. The deformation maps estimated by the proposed S-Net tend to be smoother, since the symmetric displacement map only needs half pathway, instead of a long pathway, which is easier to penalize the smoothness. Experimental results showed that our method successfully reduces the folds of estimated maps while providing more accurate registration results.

## 4. Discussion

S-Net learns for image registration tasks in an unsupervised end-to-end fashion using an image similarity metric for optimization so that the training for this S-Net does not require the known deformation field, which is difficult to obtain for medical image registration. Furthermore, we have also evaluated our framework for the number of folds with the traditional registration methods and single-direction deep-learning-based registration methods. The deformation maps estimated by the proposed S-NET tend to be smoother, since the symmetric displacement map only needs a half pathway, instead of a long pathway, which is easier to penalize the smoothness. Experimental results showed that our method successfully reduces the folds of estimated maps while providing more accurate registration results.

The total loss function in S-NET consists of two types of six losses. However, the multiple losses weight (hyperparameters) of our S-NET training is hard to balance. Therefore, we did some experiments to determine the weight of multiple losses in Figure 4. We set *α*=1 and *β*=0.01 that can achieve good performance, and after *γ* > 100, it has little effect on the results. In our experiment, we set *α*=1, *β*=0.01, and *γ*=100. It is difficult to balance multiple losses is a common problem in deep-learning-based registration methods. In future work, we hope that we can learn hyperparameters through learning.

The article "Symmetric Deformable Registration via Learning a Pseudomean for MR Brain Images" was published in 2021. Journal: J Healthc Eng.

## 5. Conclusion

We presented a new symmetric training strategy for an unsupervised deep-learning-based registration framework, which can better estimate the large local deformation during registration. In particular, we utilize a pseudomean as an intermediate target registration space, and a long deformation pathway can be divided into two short deformation pathways. Experimental results have shown promising registration performance for both accuracy and field smoothness.

## Figures and Tables

**Figure 1:** Overview of our method. Learning the parameters of S-Net by unsupervised training. The input consists of subject image *I*^*S*^, the template image *I*^*T*^ , and their difference map; the outputs are the 3D displacement maps.

**Figure 2:** The symmetric image registration scheme. (a) Illustration of the hypothesis of the symmetric image registration; (b) the whole deformation field from template to subject can be calculated by *F*=*ϕ*^*T*^∘(*ϕ*^*S*^)^−1^, and the inverse deformation field from subject to template can also be obtained by *F*^−1^= *ϕ*^*S*^∘(*ϕ*^*T*^)^−1^.

**Figure 3:** The results of the S-Net. From left to right, the column shows subject, final warped template image, middle warped subject image, middle warped template image, final warped subject image, and template image. (a) Subject image. (b) Final warped template image. (c) Middle warped subject image. (d) Middle warped template image. (e) Final warped subject image. (f) Template image.

**Figure 4:** Effect of varying the regularization parameters  *α*, *β* , and *γ* on Dice score. (a) The best results occur when *α*=1 and *β* and *γ* are fixed at 0.01 and 100. (b) The best results occur when *β*=0.01 and *α* and *γ* are fixed at 1 and 100. (c) The best results occur when *γ*=100 and *α* and *β* are fixed at 1 and 0.01. As the weight increases, the results rarely change.

**Table 1:** Dice score (%) for subject-to-subject alignment using Demons, SyN, VoxelMorph, and the proposed S-Net.

Dataset	D. Demons	SyN (CC)	VoxelMorph (CC)	VoxelMorph (MSE)	Proposed method
LPBA40	68.7 ± 2.4	*71.3* ± *1.8*	71.2 ± 2.8	71.6 ± 2.4	**71.8** ± **2.1**
IBSR18	54.6 ± 2.2	**57.4** ± **2.4**	54.2 ± 3.4	55.2 ± 2.9	*56.8* ± *2.5*
CUMC12	53.1 ± 3.4	*54.1* ± *2.8*	51.8 ± 4.1	53.1 ± 3.5	**54.4** ± **3.2**
MGH10	60.4 ± 2.5	**62.1** ± **2.4**	59.6 ± 2.9	60.2 ± 2.6	*62.4* ± *2.4*
Time (s)	114	1330	**0.31**	**0.31**	3.6

**Table 2:** Folds (|*J*_*ϕ*_(*p*)| < 0) results for subject-to-subject alignment using Demons, SyN, VoxelMorph, and the proposed S-NET. Folds refer to the average number of folds.

Dataset	D. Demons	SyN (CC)	VoxelMorph (CC)	VoxelMorph (MSE)	Proposed method
LPBA40	13.71 ± 2.91	**0**	28.52 ± 14.92	44.04 ± 13.83	*3.28* ± 0.78
IBSR18	15.59 ± 8.14	**0**	44.26 ± 15.31	67.57 ± 19.59	*7.56* ± *1.86*
CUMC12	21.02 ± 9.38	**0**	39.37 ± 11.65	48.92 ± 15.28	*7.29* ± *1.47*
MGH10	18.92 ± 6.54	**0**	42.17 ± 13.26	56.72 ± 16.76	*6.63* ± *1.53*

The article "Symmetric Deformable Registration via Learning a Pseudomean for MR Brain Images" was published in 2021. Journal: J Healthc Eng.

## Data Availability

The databases of LPBA40, IBSR18, CUMC12, and MGH10 can be downloaded from the registration grant challenge at https://continuousregistration.grand-challenge.org.
